# Efficacy of Drug-Eluting Bead Transarterial Chemoembolization in the Treatment of Colorectal Cancer Liver Metastasis

**DOI:** 10.1155/2022/4930047

**Published:** 2022-04-13

**Authors:** Sipan Chen, Yaobo Yang, Yang Jiao, Lei Hou, Hulin Chang, Sida Liu, Zhaoyong Yan

**Affiliations:** ^1^Department of Interventional Radiology, Shaanxi Provincial People's Hospital, Xi'an, China; ^2^Department of Medical Oncology, Shaanxi Provincial People's Hospital, Xi'an, China; ^3^Department of Hepatobiliary Surgery, Shaanxi Provincial People's Hospital, Xi'an, China; ^4^Department of General Surgery, Shaanxi Provincial People's Hospital, Xi'an, China

## Abstract

We aimed to investigate the efficacy and safety of drug-eluting bead transarterial chemoembolization (DEB-TACE) in the treatment of colorectal cancer liver metastasis. A total of 120 patients with colorectal cancer liver metastasis were divided into the TACE group (receiving TACE treatment, *n* = 60) and the DEB-TACE group (receiving DEB-TACE treatment, *n* = 60). At 1 month after treatment, the objective response rate (ORR) in the TACE group and DEB-TACE group were 65.0% (39/60) and 78.3% (47/60), respectively, and the disease control rate (DCR) was 78.3% (47/60) and 85.0% (51/60), respectively. Three months later, the ORRs in TACE and DEB-TACE groups were 63.3% (38/60) and 75.0% (45/60), and the DCRs were 76.7% (46/60) and 81.7% (49/60). We showed that the 1-year overall survival (OS) in TACE and DEB-TACE groups were 100% (60/60) and 88.3% (53/60), respectively, and the 2-year OS were 78.3% (47/60) and 61.7% (37/60). Further analysis indicated that the OS in the DEB-TACE group was significantly longer than that in the TACE group (*P* = 0.045). DEB-TACE is effective, safe, and feasible in the treatment of colorectal cancer liver metastasis, which can effectively improve the survival of patients.

## 1. Introduction

Colorectal cancer ranks 3rd among the most common malignancies globally, and the liver is the major metastasis site [1, 2]. According to a study, the vast majority of liver metastases of colorectal cancer patients cannot be resected radically [3]. Liver metastasis of cancer often occurs and its surgical resection rate is low, and palliative treatments have become the dominant treatment of liver metastasis, which include systemic chemotherapy, transarterial chemoembolization (TACE), radiofrequency ablation, targeted therapy, and radiotherapy. Among these therapeutics, TACE is the most commonly adopted [4, 5]. Embolization agent is one of the major factors influencing TACE. Lipiodol and chemotherapeutic drug emulsion are often adopted as embolization agents in conventional TACE (cTACE). However, liver metastasis is a type of tumor with poor blood supply, which leads to poor deposition of lipiodol. As a result, the embolization effect is not satisfactory. Drug-eluting bead (DEB) embolization uses a new type of drug-loaded microspheres that can continuously kill tumors by slowly releasing drugs [6, 7]. Studies have proved that DEB embolization shows a good treatment effect for metastatic liver cancer [8, 9].

Conventional TACE is mainly loaded with lipiodol, which is a classical embolization agent and can locate the tumor. However, it is unstable and may lead to more complications, thus affecting the efficacy [10, 11]. Meanwhile, DEBs possess the following characteristics: (1) The microspheres have a uniform and regular shape and complete particle sizes, which can better embolize tumor-feeding arteries. (2) DEBs are able to release antitumor medicine continuously and slowly in tumor tissues, which can significantly increase the drug concentration in tumor tissues and control recurrence. (3) Microspheres firmly combined with antitumor drugs can dramatically decrease the amount of medicine released into the body circulation, thus decreasing the toxic side effects of drugs [12, 13]. Currently, DEB-TACE is widely applied in primary liver cancer with satisfactory results [14]. The aim of the current research was to explore the safety and efficacy of DEB-TACE and TACE in intrahepatic metastasis of colorectal cancer.

## 2. Materials and Methods

### 2.1. General Data

The clinical data of 120 patients (with an average of 52.5 ± 9.7 years) with unresectable colorectal cancer liver metastasis admitted to our hospital were analyzed. Inclusion criteria includes (1) colorectal cancer cases with liver metastasis diagnosed according to the histological, cytological, or imaging diagnostic criteria, and the metastasis was within the liver, with measurable lesions, (2) those with hepatic neoplasm untreated by interventional therapy (TACE, ablation, iodine seed therapy, etc.) within the past 3 months, and (3) patients with Eastern Cooperative Oncology Group (ECOG) score ≤1 point and life expectancy ≥3 months. Exclusion criteria were shown as follows: (1) patients with distant metastasis besides liver metastasis, (2) those with severe liver dysfunction (Child–Pugh class C), including jaundice, hepatic encephalopathy, refractory ascites, or hepatorenal syndrome, (3) those with severe coagulation dysfunction, (4) those with completely obstructed main portal vein and less collateral vessels, (5) those with cachexia or multiple organ failure, or (6) those who cannot cooperate due to mental disorders or other reasons. Patients were divided into the TACE group (receiving TACE treatment, *n* = 60) or DEB-TACE group (receiving DEB-TACE treatment, *n* = 60). There are no statistical significances regarding the demographical data between the two groups (*P* > 0.05) (Table 1). Patients were informed before the study according to the Helsinki Declaration. This study was approved by the Ethics Committee of Shaanxi Provincial People's Hospital.

### 2.2. Treatment Methods

In the TACE group, following anesthesia, the catheter was inserted into the hepatic artery through a femoral artery puncture for angiography. After the diameter and number of tumor lesions and the feeding artery were determined, oxaliplatin (50 mg) + raltitrexed (4 mg) was injected through the artery, and the emulsion was prepared with irinotecan (80 mg) + lipiodol (10 mL). The coaxial microcatheter method was adopted for superselective catheterization of the responsible feeding artery, and the embolization drugs were slowly infused until reaching the peripheral embolization level, followed by extubation. The above treatment was repeated once every 3–4 weeks, with a total of 2 treatments. In the DEB-TACE group, the configuration of perfusion drugs was the same as that in the TACE group. The HepaSphere DEBs (50–100 *μ*m in diameter, twofold configuration, Merit Medical Systems, Inc.) were slowly infused into the tumor notorious vessels through the catheter. The same systemic treatment was performed in both groups.

### 2.3. Observation Indexes

At 1 and 3 months after treatment, the curative effect was evaluated according to the modified Response Evaluation Criteria in Solid Tumors (mRECIST), which was divided into complete remission (CR), partial remission (PR), stable disease (SD), and progressive disease (PD). The objective response rate (ORR) was defined as CR + PR, and the disease control rate (DCR) was defined as CR + PR + SD. Adverse reactions and related medications during follow-up were recorded. Adverse reactions were assessed according to the National Cancer Society Common Toxicity Standard CTC4 [15]. The survival of patients was recorded during follow-up, which ended in May 2021.

### 2.4. Statistical Analysis

Statistical Product and Service Solutions (SPSS) 22.0 was utilized for statistical analysis. Measurement data were expressed as mean ± standard deviation (‾*χ* ± *s*) and compared by *t*-test between groups. Chi-square was employed for comparisons of the enumeration data between groups. *P* < 0.05 indicated a statistically significant difference.

## 3. Results

### 3.1. Analyses of Clinical Efficacy

In the TACE group, there were 0 cases of CR, 39 cases of PR, 8 cases of SD and 13 cases of PD, with an ORR of 65.0% (39/60) and DCR of 78.3% (47/60). In the DEB-TACE group, there were 1 case of CR, 46 cases of PR, 4 cases of SD, and 9 cases of PD, with an ORR of 78.3% (47/60) and DCR of 85.0% (51/60). The curative effect was evaluated again at 3 months after treatment. The ORR and DCR were 63.3% (38/60) and 76.7% (46/60), respectively, in the TACE group, while the ORR and DCR were 75.0% (45/60) and 81.7% (49/60), respectively, in the DEB-TACE group. There was no statistical significance regarding the ORR and DCR at 1 and 3 months after treatment (*P* = 0.156, *P* = 0.480, *P* = 0.235, *P* = 0.654, Table 2).

### 3.2. Analyses of Side Effects

Side effects mainly included abdominal pain, fever, nausea and vomiting, diarrhea, fatigue, liver function damage, leukopenia, anemia, and thrombocytopenia, which were mainly grade I-II, and the symptoms were improved. No grade IV toxicity and no progressive disease or death related to adverse reactions occurred in both groups. The incidence rate of abdominal pain in the DEB-TACE group was significantly higher than that in the TACE group (51.7% *vs.* 30.0%, *P* = 0.025). The incidence of leukopenia was significantly lower in the DEB-TACE group than that in the TACE group (8.3% *vs.* 28.3%, *P* = 0.008). The incidence rate of anemia in the DEB-TACE group was 18.3%, which was remarkably lower than 43.3% in the TACE group (*P* = 0.005). The incidence rate of thrombocytopenia was 10.0% in the DEB-TACE group, which was significantly lower than 33.3% in the TACE group (*P* < 0.001). In addition, the incidence rate of liver function damage in the DEB-TACE group was 26.7%, which was significantly lower than 55.0% in the TACE group (*P* = 0.003) (Table 3).

### 3.3. Follow-Up Analyses

The 1-year OS were 100% (60/60) in the TACE group and 88.3% (53/60) in the DEB-TACE group, respectively. The 2-year OS were 78.3% (47/60) and 61.7% (37/60), respectively. The survival curves of the two groups of patients were plotted using the Kaplan–Meier method. Further analyses manifested that the OS in the DEB-TACE group was significantly better than that in the TACE group (*P* = 0.045) (Figure 1).

## 4. Discussion

According to a previous report, 15 patients with colorectal cancer liver metastasis were treated with irinotecan-eluting beads (DEBIRI)-TACE, their progression-free survival (PFS) and OS were 8 months and 13 months, respectively, and one of the patients whose liver metastasis was reduced so that surgical resection was feasible [16]. In the study of Iezzi et al. [17], 20 patients with colorectal cancer liver metastasis were treated with DEB-TACE, and the PFS and OS were 4 months and 7.3 months, respectively [17]. To compare the efficacy of DEB-TACE with that of FOLFIRI (irinotecan + fluorouracil + calcium folinate), Fiorentini et al. [18] enrolled 74 patients with colorectal cancer liver metastasis in their study, and the results showed that the PFS and OS were longer, and the systemic adverse reactions were less in the DEB-TACE group than those in the FOLFIRI group. Akinwande et al. [19] showed that FOLFOX combined with DEBIRI dramatically prolonged the survival time of patients. In addition, Cucchetti et al. [14] found that DEB-TACE could shorten the hospital stay and improve life quality. Vogl et al. [20], reported 224 patients with liver metastasis treated with DEB-TACE and found that DEB-TACE could reduce the diameter of liver target lesions by 21.4% on average, showing a statistically significant difference (*P* < 0.05). Martin et al. [21] retrospectively analyzed 55 patients receiving DEB-TACE and found that the ORR was 66% at 6 months and 75% at 12 months, and the OS and PFS were 19 months and 11 months, respectively. According to Martin et al. [22], postembolization syndrome accounted for 40–63% of all adverse reactions. Stutz et al. [23] found that abdominal pain (59.3%) was the most common adverse reaction of patients after DEB-TACE treatment. Various study results revealed that DEB-TACE can benefit the survival of patients while bringing no obvious intolerable toxic and side effects, and postembolization syndrome is the major adverse reaction.

In this study, the treatment effect of 60 patients with digestive tract tumor liver metastasis treated with DEB-TACE was compared with that of 60 patients treated with cTACE. The follow-up analysis manifested that OS in the DEB-TACE group was superior to that in the TACE group (*P* = 0.045). In addition, it was found that postembolization syndrome was the major common adverse reaction of patients in the DEB-TACE group, mainly manifested as fever, abdominal pain, nausea and vomiting, etc. The causes of fever and abdominal pain were ischemia and necrosis of local tissues after hepatic artery embolization, and nausea and vomiting were associated with chemotherapy drugs. In the present study, 26 patients (43.3%) in the DEB-TACE group had grade I-II abdominal pain, which was tolerated by all patients, and another 5 patients (8.3%) had grade III abdominal pain, which could be alleviated after being treated with opioids. The incidence of postoperative fever (fluctuating around 38.5°C) was 31.7%, and there was no high fever (>39°C). Besides, the above postembolization syndrome of the patients was recovered after about 1 week. By the end of follow-up time, no severe complications such as bleeding at the puncture site and liver and kidney failure occurred in the DEB-TACE group [24].

However, limitations still existed in this retrospective study. The limited sample size and short and incomplete follow-up weakened the evidence level. Therefore, the conclusion in this study needs to be further verified through large-sample multicenter long-term follow-up studies in the future.

## 5. Conclusion

DEB-TACE is effective, safe, and feasible in the treatment of colorectal cancer liver metastasis, which can effectively improve the survival of patients.

## Figures and Tables

**Figure 1:** The survival analysis of the patients in the 2 groups. The overall survival rate in the DEB-TACE group was superior to that in the TACE group (*P* = 0.045).

**Table 1:** Demographics and general clinical data of all studied patients.

Parameters	TACE group	DEB-TACE group	*P* value
	*n* = 60	*n* = 60	
Gender (male/female)	37/23	32/28	0.460
Age (years)	51.59 ± 9.47	53.18 ± 9.84	0.369
Primary tumor			0.574
Colon	35 (58.3%)	39 (65.0%)	
Rectum	25 (41.7%)	21 (35.0%)	
Number of liver tumors			0.447
Single	19 (31.7%)	24 (40.0%)	
Multiple	41 (68.3%)	36 (60.0%)	
Largest tumor diameter (cm)	10.28 ± 2.56	10.56 ± 2.61	0.554
Child–Pugh grading			0.562
A	42 (70.0%)	38 (63.3%)	
B	18 (30.0%)	22 (36.7%)	
ECOG (points)			0.693
0	17 (28.3%)	20 (33.3%)	
1	43 (71.7%)	40 (66.7%)	

**Table 2:** Analyses of clinical efficacy.

	TACE group *n* = 60	DEB-TACE group *n* = 60	*P* value
1 month postoperative			
CR	0 (0%)	1 (1.7%)	
PR	39 (65.0%)	46 (76.7%)	
SD	8 (13.3%)	4 (6.7%)	
PD	13 (21.7%)	9 (15.0%)	
ORR	39 (65.0%)	47 (78.3%)	0.156
DCR	47 (78.3%)	51 (85.0%)	0.480
3 months postoperative			
CR	0 (0%)	1 (1.7%)	
PR	38 (63.3%)	44 (73.3%)	
SD	8 (13.3%)	5 (8.3%)	
PD	14 (23.3%)	11 (18.3%)	
ORR	38 (63.3%)	45 (75.0%)	0.235
DCR	46 (76.7%)	49 (81.7%)	0.654

**Table 3:** Analyses of side effects.

	TACE group *n* = 60	DEB-TACE group *n* = 60	*P* value
Abdominal pain	31 (51.7%)	18 (30.0%)	0.025
Fever	19 (31.7%)	15 (25.0%)	0.517
Nausea and vomiting	23 (38.3%)	20 (33.3%)	0.416
Diarrhea	24 (40.0%)	14 (23.3%)	0.077
Fatigue	25 (41.7%)	15 (25.0%)	0.081
Leukopenia	17 (28.3%)	5 (8.3%)	0.008
Anemia	26 (43.3%)	11 (18.3%)	0.005
Thrombocytopenia	22 (33.3%)	6 (10.0%)	0.001
Liver function damage	33 (55.0%)	16 (26.7%)	0.003

## Data Availability

The datasets used and analyzed during the current study are available from the corresponding author on reasonable request.
